# Filtering Inequality: Screening and Knowledge in Senegal’s Topography of Hepatitis B Care

**DOI:** 10.3389/fphar.2020.561428

**Published:** 2021-04-12

**Authors:** Noemi Tousignant

**Affiliations:** University College London, London, United Kingdom

**Keywords:** Senegal, Hepatitis B, access to treatment, inequalities in access to healthcare, ethnography

## Abstract

Only a fraction of the estimated tenth or so of Senegalese who are chronically infected with hepatitis B virus (HBV) have been diagnosed. Of these, few have been assessed for their risk of progressing to potentially fatal liver disease (indicating need for treatment), and fewer still are taking antiviral drugs. A massive gap between those needing and getting treatment is widely acknowledged among experts. But given that HBV and its biomedical treatment options are largely invisible in bodies, health data, care practices, public messaging, or mass media, how can we observe, ethnographically, the effects of constraints on and inequalities in treatment? What are the stakes of access to drugs, when this access is not being sought out, claimed, or enacted? This article tackles these questions by examining how HBV is being enacted in Senegal, but not necessarily in relation to antiviral treatment. I first describe the emergence, over the past decade and a half, of an exclusionary topography of HBV diagnosis and treatment. I introduce the notion of “filtration” to describe the effects of this topography on the formation of potential “subjects of access.” The diagnostic therapies and expertise required to determine need for treatment are expensive, urban, and largely privatized. Moreover, knowledge about HBV and its possibilities of care circulates in narrow and sparsely distributed channels. Only a tiny minority of persons are effectively “filtered into” care, while issues of access remain largely outside of public debate. I then move onto small-scale efforts, led by rural primary health workers and community associations, to raise awareness of and expand screening for HBV. Those driving information and screening either do not reveal that effective drugs exist or locate these beyond the reach of most of their audiences or patients. Why then do they do it? I examine the logics and effects of their work to identify the forms of inclusion, care, efficacy, and explanation these open up. At the same time, I seek to discern the indirect effects of unequal access to knowledge and resources in the ambivalence, uncertainties, and contradictions that pervade these efforts to inform, diagnose, and advise.

## Introduction

“We have accessibility,” said an infectious disease specialist as she opened the hepatitis B virus (HBV) session of a 2019 research meeting in Dakar. Quickly, she caught and corrected herself: “well, in any case, availability.”

This slip states a seemingly obvious point: drugs “being there” is not the same as drugs getting to all those who need treatment. But how are we to identify those whose lives are marked by the gap between available drugs and their accessibility as HBV treatment? Public health discourse generally assumes that the potential subjects of HBV treatment are *already* out there, even if they are asymptomatic, as chronic HBV infection often is. They need only to be diagnosed. Identifying virus carriers requires a serological test for hepatitis B surface antigen (HBsAg). Not all carriers, however, are or will *ever* get sick from their infection. Current consensus is that only those at higher risk of developing severe, usually fatal cirrhosis and cancer should be treated. Identifying these treatment candidates requires further diagnostic testing and interpretation of viral activity, liver damage, and other indicators of risk.

Population infection rates estimated from sample surveys suggest that the majority of the world’s HBV carriers are not diagnosed or linked into care, that is, effectively referred for treatment eligibility assessment followed by prescription and/or monitoring. Global advocacy for access to HBV treatment, which has emerged in and around the World Health Organization (WHO) and World Hepatitis Alliance (WHA) in the past decade, has focused on improving and demonstrating the feasibility of large-scale screening and assessment in resource-poor settings, where most HBV carriers live. Although drug prices and supply certainly remain a concern, the wide availability of generic antivirals for HBV (notably tenofovir disoproxil fumarate) has shifted attention to diagnosi*s*. The experts convened to develop and review the WHO’s first treatment guidelines, published in March 2015, focused in particular on developing diagnostic pathways that bypassed the high-cost equipment and expertise—including HBV-DNA quantification (i.e., PCR-dependent viral load testing), liver ultrasonography and specialist consultations—on which assessment protocols used in high-resource settings depend (WHO, 2015). The WHO also issued recommendations on screening strategies in different epidemiological settings, included where infection is widely distributed across the “general” population rather than concentrated in “high risk” groups (WHO, 2017). For public health, disparities between the massive number of people assumed to be infected and the much lower numbers who are screened, referred, and treated pose problems of *efficacy* (unprevented future morbidity and mortality) and of *equity* (exclusion from potentially life-saving treatment).

For ethnography, however, the scarcity of HBV diagnosis also poses a methodological problem, especially given the variable and delayed perceptibility of an infection that often remains asymptomatic or only vaguely symptomatic for most or all of carriers’ lives.

Who are the potential subjects of HBV treatment, and how are they constituted as such? Where can we locate the gap between available treatment and its accessibility to those who have not or only partially been constituted as its subjects? How does this gap manifest around the limited and uneven presence of embodied and diagnostic knowledge as well as public communication and debate about HBV infections, pathology, and care?

In Senegal, HBV screening is performed systematically and for free only to donated blood,^1^ although it is also part of the standard bundle of prenatal tests and thus is increasingly offered for a fee to pregnant women across the country. The equipment and expertise needed to assess treatment eligibility are concentrated in urban areas and are mostly available through private practice and test sites, or fee-paying services in teaching hospitals.

Moreover, public talk about HBV and its treatment—as advocacy, health messaging, or news coverage—is sparse. “Awareness-raising” has been small in scale as well as episodic. Examples include media coverage of a few, high-profile conferences on hepatitis held in Dakar as well as of annual “World Hepatitis Day” events. There are also occasional hepatitis-themed features or episodes, many serving as publicity for “neo-traditional” healers, on radio, television or internet channels. There have been no mass campaigns to inform that HBV infection is very common among unvaccinated adults (more than one in ten for those born before 2005) and can lead to fatal disease. Nor is information widely available about how and where HBV infection can be diagnosed, assessed, and treated. A qualitative study in rural Senegal found that only a third of nonexperts had ever heard of “Hepatitis B” (Boye et al., 2020). This study, and other questionnaire-based research, also points to gaps in the knowledge of healthcare practitioners such as nurses and generalist physicians, (Lawson et al., 2017; Jaquet et al., 2017a, b; Djaogol et al., 2019), suggesting a lack of investment in training. Many are thus unlikely to prescribe screening tests or refer for assessment.^2^ In 2019, many experts in Senegal questioned the robustness of available seroprevalence data, and viral hepatitis was just being integrated into the national disease surveillance and reporting system. HBV thus has limited visibility not only as a bodily experience and as a test result, but also in clinical training, advice, and practice; in epidemiological data; in public health messaging; and in media coverage.

Given this invisibility, how is it possible to engage with inequalities in access without assuming that its potential subjects are “already out there,” existing biologically by their (undiagnosed) viral infection and immune response? In this article, I propose to begin, empirically, by examining how HBV is being enacted in Senegal but *not necessarily as a condition for antiviral treatment.* I focus on the practices that bring HBV into being an object of knowledge and care in three types of settings, which form the core sections of this article: urban specialized HBV care, where treatment eligibility assessment followed by prescription are offered; the screening and advice provided by primary healthcare workers in one rural district; and two sets of “grassroots” initiatives to create collective awareness about HBV.

## METHODS AND APPROACH

This article is based on fieldwork I conducted in Senegal in 2019. My broader research project concerns how aetiological knowledge about liver cancer has been produced and deployed in West Africa from the 1950s to the present. Given that chronic HBV infection was shown to be a risk factor in the 1970s–1980s and that antiviral drugs are, since the late 1990s, recognized to prevent infection-induced liver damage (cancerous and cirrhotic), my research included an ethnographic focus on HBV care in Senegal.

The three core sections of the article draw, respectively, on interviews and conversations with HBV specialists and experts; primary healthcare (PHC) workers in the rural health district of Nioro; and laypersons active in HBV screening and communication. The first group comprises approximately 20 internists, gastroenterologists, infectious disease specialists, epidemiologists, and virologists, mostly based in the capital city of Dakar. This covers a significant portion of the persons actively involved in HBV research and care in Senegal. I also attended several meetings on HBV care and research as well as conducted an extensive review of published research, policy documents, and media coverage. In February-March and July 2019, I spent four nonconsecutive weeks in Nioro, which is located in south-central Senegal between the regional capital of Kaolack and the Gambian border. I selected it on the basis of anecdotal reports of high liver cancer incidence, as well as its association with peanut consumption and farming given the identification of aflatoxin, a common contaminant of peanuts, as a cofactor of liver cancer. I interviewed 25 primary healthcare workers, including 11 nurses who managed village-level health posts (*infirmier chef de poste*, or ICP), 4 retired ICPs who had opened private clinics, and 10 midwives. A research assistant, Aissatou Diouf, was present during some interviews and participated in discussions. I also spoke with a range of other health actors at community, district and regional levels. Finally, I sought out and interviewed individuals who I heard had initiated HBV information and screening activities.

The interviews were semistructured and covered the history, practices, itineraries, landscape, and challenges of care provision for patients with HBV infection, liver cirrhosis, and cancer. They were either recorded or extensive notes were taken. All informants were provided with written and oral information about the project and gave explicit consent to participate and for interviews to be recorded (or not) and cited. Research authorization was also obtained in Senegal at national, regional, and district levels. Participants are systematically anonymized in this article, except for public figures who also agreed for interview content to be cited.

### The Ethnography of Access to Treatment in Africa: Visibility and Inequality in HIV and HBV

Access to treatment has been a core focus of the anthropology of HIV/AIDS in Africa. From the late 1990s to the mid-2000s, antiretroviral drugs (ARVs) were available in limited quantity through private and personal channels, as well as in research trials and pilot treatment projects. Anthropologists revealed the effects, not only on bodies and survival, but also on social relations, political debate, and moral deliberation, of these uneven provisions and of the inequalities they generated. Nguyen (2010), for example, traced how, in Burkina Faso and Côte d’Ivoire, the performance of HIV-positive identities through associational involvement and public testimonials enabled some to gain access to scarce drugs, yet also gave rise to collective claims to treatment as a right based on a biological condition. At a moment when ARVs were getting cheaper in Uganda and being piloted in treatment programs, yet remained beyond reach for the majority, Whyte et al. (2004) described how unequal access created moral dilemmas and social tensions in clinical practice, family relations, and public debate. Desclaux et al. (2002) and Desclaux (2004) observed the effects of drug fees on patients enrolled in Senegal’s pioneering public treatment program. They noted that even subsidized and sliding rates created inequality at two levels: in the affordability of treatment and in the burdens that finding money for treatment imposed on patients, who had to disclose their status in order to activate solidarity networks.

This body of work is rich in insights about the politicization of access and the subtle tensions and fault lines that treatment inclusion and exclusion can (re)produce. Such insights can guide the questions we pose about access to HBV care in Africa. Yet there are important differences in how HIV and HBV have been made visible as a threat to bodies, lives, and society, and as being treatable by antiviral drugs (even though some of the same molecules are used against both viruses). The prospect of ARV treatment increased and modified the visibility of HIV, for example through test uptake and disclosure of status. Yet ARVs entered into landscapes where HIV/AIDS had already been given a palpable presence through, for example, rumors of suspicious deaths (Fassin 1994), prevention campaigns that figured mass education and screening (with counselling, see Whyte et al., 2018), and patient associations, testimonies, and activism (Robins and Lieres, 2004; Nguyen, 2010).

Around what kinds of visibilities of HBV infection and care can we observe the effects of treatment (in)accessibility and its inequalities? There have been few qualitative or ethnographic studies of HBV in Africa (or elsewhere), with the exception of revealing but nonextensive studies in Côte d’Ivoire (Pourette and Enel, 2014), Burkina Faso (Giles-Vernick et al., 2016; Giles-Vernick and Hejoaka, 2020), Cameroon (Chabrol, 2018, 2019; Chabrol et al., 2019), and Senegal (Boye et al., 2020). These point to the challenges to access posed by the high cost of further HBV care and lack of knowledge about HBV among both laypersons and health workers. They also show that the limited spaces and moments when HBV is made visible, for example when a diagnosis is made after blood donation, are located within topographies and trajectories marked by uncertainty about the meaning of infection and its invisibility as a collective presence (especially Giles-Vernick and Hejoaka, 2020; Chabrol, 2018, 2019). Building on this work, I seek to discern the *indirect* effects of the limited visibility of HBV and of access inequalities on broader (but far from universal) provisions of HBV diagnosis, information, and care.

I begin by mapping out the equipment, drugs, and expertise through which antiviral therapy is provided in Senegal. Yet I also attend to how the privatization of both specialized HBV care and communication limits the visibility of treatment beyond the narrow, urban, and exclusive circuits through which drugs and eligibility assessments can be accessed. In the following two sections, I turn to spaces where screening tests are performed, namely, in rural primary healthcare and through community action, but generally *not* in view of initiating trajectories into specialized assessment and treatment. Rather than dismissing testing without “linkage to care” as a therapeutic dead-end, as a public health perspective might, I propose to attend to these efforts as enactments of HBV with their own logics and effects. These open up unexpected forms of inclusion, care, efficacy, and explication that bypass inaccessible assessment and treatment. At the same time, these efforts are shaped by uneven distributions of information about HBV and other resources for care, and some of their actors are troubled by the restrictions on access to treatment they know or suspect lie beyond.

## Results

### A Historical Topography of “Availability”

Most specialists trace the first expansion of HBV treatment in Senegal to a trial, “HEPADAK,” initiated in 2003. Subjects were provided with access to manufacturer-donated lamivudine.^3^ Before this, a handful of Senegalese purchased the less effective pegylated interferon abroad or in downtown Dakar, at the country’s best-stocked private pharmacy. HEPADAK subjects were enrolled by specialists in four Dakar hospitals and private clinics (Vray et al., 2006), who were referred as HBV infected individuals by major blood banks. Confronted with difficulties in using biopsy to assess liver damage, project researchers negotiated additional funding to purchase and evaluate a trademarked liver ultrasonograph, a portable and noninvasive imaging technology, in Dakar (Mbaye et al., 2011). After the trial, the machine was made available at a cost to patients of 60,000 CFA/106 USD per test (until it broke down).

Trial researchers and the funder, a French public research agency, were committed to ensuring posttrial access to lamivudine. Negotiations with the Ministry of Health and National AIDS program allowed HBV patients to “dip into” donor-purchased stocks of HIV drugs, switching from lamivudine to tenofovir (both used for HIV) in 2010.^4^ That such an arrangement was possible suggests that the number of individuals in specialist HBV care was low at the time and grew slowly afterward. The availability of HIV drugs for HBV patients does not seem to have been widely advertised (one specialist assured me it was not “a secret,” but others noted the need to avoid donor scrutiny). In any case, even if the drugs were free, a full assessment of treatment eligibility cost, before 2014, upward of 150,000 CFA/264 USD, with tests to be repeated every six to twelve months for monitoring.^5^ By 2014, however, HBV patients were blamed for causing ARV stockouts (Dakaractu, 2014). Still, as late as the end of 2017, it was estimated that only 893 individuals were taking drugs for HBV in Senegal (Programme National de Lutte contre les Hépatites, 2018).^6^

The cost of HBV treatment was briefly but forcefully put in the spotlight in the Senegalese media in 2011–2012. Having focused on vaccination since 1998, the country’s pioneering National Hepatitis Program (PLNH), established by Aminata Sall Diallo, organized a high-profile pan-African meeting in Dakar to mark the first “World Hepatitis Day” in July 2011 (Sall Diallo, 2018). The conference issued a collective call to action, the “Appel de Dakar,” which, notably, pleaded for drug price reductions (Sall Diallo, 2012). Sall Diallo also encouraged an articulate former soldier, Ibrahima Gueye, to speak out about his struggles to pay for treatment (e.g., Diatta, 2015a) and to form the patient association *Saafara Hépatites* in late 2011. Speaking to the media, which gave wide coverage to PLNH-organized 2012 World Hepatitis Day events, Sall Diallo and Gueye denounced the “excessive,” “out-of-reach” and “horribly expensive” price of HBV drugs (e.g., RTS 2012; 2STV 2012; Senewebdirect 2012). However, the figures they gave were for pegylated interferon, which Gueye had been prescribed because of a coinfection with HBV (hepatitis “delta,” a virus that requires HBV to replicate), and which was sold only by the best-supplied private pharmacies for 159,000 CFA/280 USD per week (a full course lasting a minimum of 48 weeks). They did not mention tenofovir, which was available in generic form, nor the fact that some HBV patients were already obtaining these from the HIV program.

Meanwhile, around 2012, the PROLIFICA study, which was the first to evaluate the feasibility of large-scale test-and-treat strategies in Africa with a view to informing strategies and advocacy for expanded access, was launched in various sites (Allain, 2016; Howell et al., 2016). One of these was Thies, a regional capital just over an hour’s drive (without traffic) from Dakar. Unlike HEPADAK, which had collected subjects through existing, limited channels of diagnosis and care, PROLIFICA set up “community” screening in workplaces and villages. It also brought some diagnostic services and drug distribution beyond the capital, notably setting up a second liver ultrasonography machine (Touré et al., 2017; Cohen et al., 2019). Patients outside the trial could be assessed with the latter for 10,000 CFA/18 USD. The number of trial subjects enrolled, however, was relatively low: in 2019, a researcher spoke of a follow-up cohort of 460.

HBV-DNA testing capacity was set up in Dakar in 2013 or 2014. One machine was obtained by a military pharmacist, involved in research, who told me he had witnessed the “suffering” of patients from the high price and long wait associated with shipping samples for testing in France. So, he told me, he approached a PCR manufacturer and pleaded with them: “I’m passionate about hepatitis B, but [you] have to help us, give us the apparatus.” They did, but operating costs, he says, mean he needs to charge 25,000 CFA/44 USD per test in the semiprivate lab he runs. Around the same time, the Dakar Pasteur Institute, a research institution that also provides private diagnostic and vaccination services, began offering HBV-DNA tests for 35,000 CFA/62 USD. In late 2016, the regional rep of a major European diagnostics firm announced the donation of a molecular testing platform (said to cost 120 M CFA: Diatta, 2016) to the Bacteriology–Virology Laboratory of *Hôpital Le Dantec.* The rep explicitly framed this as a private initiative to fill an accessibility gap in partnership with the public sector and was able to negotiate a price of 15,000 CFA/26 USD per test (he hoped subsidization would reduce this). In the first months of 2019, however, testing had stopped due to a reagent stockout. I heard that the rep held a monopoly on the supply of kits specific to the donated apparatus and had been too busy with politics to renew the order. At one meeting I attended, this donation-supply arrangement was criticized not only for failing HBV patients, but also for bypassing public procurement rules.

Even with these price drops, viral load testing is still seen by Senegalese experts as, in their words, the “bottleneck” or “Achilles’ heel” of HBV care. This is generally the case in low-resource settings. Avoiding viral load testing, as well as expensive liver assessment such as ultrasonography, was an explicit goal in the development of WHO treatment guidelines (WHO, 2015). This reflected an explicit prioritization of a “public health approach” by which viral and liver assessment can be scaled up through simplification of tests and criteria and standardization of decision-making algorithms so that they can be used by nonspecialists.

Following this lead, the PNLH organized a meeting of Senegalese HBV experts circa 2015 with the goal of agreeing on a “national consensus” on testing, referral, and assessment protocols. This would enable the decentralization of HBV care beyond Dakar and major urban centers. By all accounts that I heard, the process failed. Some told me tensions arose between clinically oriented internal medicine specialists accustomed to working in hospital and private settings and infectious disease specialists who advocated for a public health approach modelled on HIV treatment. Whatever the reason, several meeting participants told me no agreement had been reached. A “national consensus” was published by the PNLH as a booklet but was never distributed (few knew of its existence).

In 2019, I heard many HBV experts in Senegal express doubts about the extent to which “gold standard” diagnostic assessment (such as used in high-resource settings) could be simplified and cost reduced. Many said they tried to “adapt,” but that, as one hospital specialist exclaimed: “there are norms!” Some specifically questioned the WHO’s “no-viral-load” criteria, which they thought would miss too many patients who needed treatment (see also Béguelin et al., 2018; McMahon and Dusheiko, 2018). Interviews, and the test prescriptions I have seen, indicate that most Senegalese specialists consider viral load measurement to be essential and that they often request a long list of both routine and harder-to-obtain tests. The cost of these tests adds up quickly: Gueye estimates a full assessment can cost from 100,000 to 300,000 CFA/175 to 350 USD, while the PLNH gives lower figures of 45,000–80,000 CFA/78–141 USD, probably for a “simplified” assessment (Programme National de Lutte contre les Hépatites, 2018).

In 2017, public drug procurement specifically for HBV treatment became operational as a result of negotiations between HBV specialists (including the PNLH) and the national pharmacy. The availability of this “HBV” tenofovir and its subsidized price of 5,000 CFA/9 USD for a month’s supply was, as reported in a brief newspaper item, announced by the Minister of Health “on the sidelines” of a ceremony for the reception of four donated ambulances (Ndieng, 2017). I did not see any posters, pamphlets or webpages, whether in health facilities (including the national blood transfusion center, where many get diagnosed) or the PNLH website, providing information on where to get HBV tests, consultations, or drugs. Thus, persons diagnosed as HBV-positive are dependent on referrals to specialists (and on the information these specialists will then give them) and on personal networks. I came to participate in these by advising acquaintances who tested positive for HBV, but who had not been told where or why to obtain further care. Some may learn about *Saafara Hépatites* from the news, a specialist or the hospital blood bank with which the association works. Gueye, who has parted ways with the PNLH, fields frequent calls from patients who have not been told where to get various tests, what they are for, or what the results mean. He tries to keep up to date on test prices, drug stocks, and equipment breakdowns. Specialists say their HBV caseloads are growing due to increase in referrals from blood banks as well as, more recently, from prenatal care providers. I asked one whether he thought the availability of medicines was drawing people into HBV care. “No,” he quickly answered, “I don’t think people know.”

In meetings and interviews I attended, the cost to patients of antiviral drugs was *not* a major topic of conversation. A couple of specialists admitted that it was still high “relative to incomes,” and that a handful of patients resented the shift from free to fee-paying drugs. Most, however, insisted that patients were “willing to pay” out of fear of getting liver cancer (a painful and rapidly fatal condition some may have witnessed in kin and neighbors). By contrast, I heard many express concerns about the lack of “communication” or “awareness-raising” about HBV. Some criticized the PNLH in private for its failure to do mass awareness-raising and screening, as well as to decentralize HBV care (beyond Dakar). Gueye has, in recent years, been openly critical of the program and of Sall Diallo’s autocratic leadership: “there is only her,” he said on TV (Dakar Matin, 2018; see also: Diatta, 2018). In response, Sall Diallo (2018) published an open letter detailing the program’s history of tiny budgets (currently at 27 M CFA/48 K USD, and only 36 M CFA/63 K USD at its highest point).^7^ This is the reason, she explains, why she has been forced to do all the “communication” herself: “to the extent that (my) image has been systematically associated with the fight against hepatitis in Senegal.” In an earlier interview (Diatta, 2015b), she pointed out that donors fund mass communication about HIV/AIDS, malaria, and tuberculosis but not hepatitis. Because of this “global health governance,” she has been left on her own to communicate about hepatitis “on television, on the radio, speaking to the written press. You all know me through these media.” Thus, she implies, only the diseases that donors identify as priorities can become, through mass action, matters of public health. Meanwhile, her underfunded program and its target diseases remain associated with a thin and highly personalized presence in the public arena.

Colleagues in Senegal familiar with the history of HIV activism are mystified by the absence of vocal demands for free HBV care. But this lack of mobilization may, at least in part, be a product of the topography of care that has emerged from fragmented research, personal, and commercial initiatives and in the absence of public strategies and channels for distributing knowledge (from education about infection risk to systematic screening and referral practices) about HBV and HBV care. In this topography, potential subjects of HBV treatment are constituted, or not, by being “filtered” into or out of narrow circuits of care.

I propose filtration as an extension of Nguyen’s use of triage (2010) to describe the paradoxical effects of limited ARV provision, whereby humanitarian efforts to “save lives” sort out those who may live from those left to die. Triage describes the selective allocation of scarce technologies (diagnostic and therapeutic), which, in the case of HBV care, is underpinned by the combination of high cost, urban concentration, and privatization. Some services are offered in private clinics and labs, while even in public institutions, patients are expected to bear a large portion of the costs of tests (which often depend on commercial technologies) and drugs, a fact that specialists largely accept as the normal state of affairs. By introducing filtration, I also want to draw attention to the additional, or rather amplifying, effects of sparse and uneven distributions of information and knowledge about HBV, whose channels are also, in a way, privatized. Communication about HBV is, due to lack of funding for awareness-raising, training, or even patient orientation, concentrated around public figures such as Gueye and Sall Diallo, or left to the initiative of individual practitioners. It is therefore highly personalized and small in scale. The result is that neither scarcity nor its modes of rationing have become topics of public or professional debate.

Filtration is a mediated process, in which potential subjects of treatment, their kin and clinicians, give advice and make decisions on the basis of incomplete and heterogeneous knowledge of the stakes of infection and the possibilities of care. In this mediation, obstacles such as cost, distance, and lack of knowledge are difficult to clearly delineate and may be impossible to disentangle. Some who may be able to arrange, even if at considerable sacrifice, to pay for lifesaving drugs are uninformed of their condition or of how it can be managed. Practitioners, some of whom are poorly informed about available treatment options, may selectively mete out such information to avoid futile, interrupted quests for care. What does seem clear is that filtration increases the likelihood that those to whom drugs are eventually prescribed—after having been successively filtered into care by screening, persuasive and well-informed referral and full assessment, as well as ability to pay and travel—will in fact be willing to pay for them. Meanwhile those who have been filtered *out* of care and who have not been (fully) enacted as subjects of treatment (or even of HBV) are unlikely to demand access or to criticize its inequalities. In the following section, I examine how filtration is initiated at points of primary healthcare, in a rural area where HBV screening tests are expanding yet very few are referred for assessment and treatment.

### Lateral Care

“I like hepatitis B too much!” exclaims Dr. T. “I mean I like the follow-up of hepatitis B, not,” he clarifies, laughing, “the patient.” Dr. T. is not a doctor but the nurse who heads a rural health post (ICPs are commonly addressed as “doctor”) in the district of Nioro, which is near the Gambian border and whose main town is about an hour’s drive from the regional city of Kaolack. He is describing his plan to set up a system to register and monitor his HBV patients, as he did for diabetes and hypertension. He also describes previous HBV initiatives.

In 2013–2014, during a community health education project for malaria, he “integrated”—a deliberate term of contrast with “vertical” disease-specific actions—hepatitis B (alongside diabetes and hypertension) in a series of public events such as conferences and plays. As the demand for HBV screening increased, Dr. T., again as a “personal initiative,” procured a stock of rapid tests for his health post from the District Health Centre’s Laboratory. He also organized blood drives, primarily as an HIV-screening strategy—which the district mandated each post to develop—but with the knowledge donor blood would also be tested for HBV.

Among Nioro’s PHC workers, Dr. T. appears as exceptionally enterprising; the only one to report having organized information and screening events (although another midwife-ICP pair said they had planned similar activities). Yet he was not the only one to be concerned about HBV. HBV screening is increasing in the district, as a result of occasional blood drives organized by youth or religious associations and its recent routinization in prenatal testing. The high proportion of positive results has made the infection visible as a public health problem to many PHC workers.^8^ Most ICPs have also experienced the heavy emotional burden of diagnosing or providing end-of-life care to patients with advanced liver disease. This explains, in part, why some ICPs, like Dr. T., are keen to expand screening and some midwives think it is important to persuade women to pay for a prenatal HBV test. But where does screening lead? Below I describe how practitioners, in their words, advise patients who test positive. I first examine whether and how they refer for further care, noting, in particular, their expressions of *ambivalence* about the uncertain benefits, or the high costs, of additional consultations, testing and treatment. Instead of, or alongside, referrals, PHC workers nearly always provide advice for self-care, mainly through diet. I explore this dietary advice as a form of *lateral care*, a term of contrast with the public health model of a “continuum of care”—from screening through referral, further assessment, treatment, and/or monitoring, or palliative care—that supposes a linear trajectory organized around access to diagnostics and drugs. Nonreferral and dietary advice are lateral in the sense of eschewing options that PHC workers are either poorly informed about or know to be unaffordable to the majority of their patients. Yet they also manifest preventive logics anchored in situated understandings of available resources, social relations, emotional care, and liver cancer aetiology. In concluding this section, I reflect on how lateral care both responds to and reproduces inequalities in patients’ capacity to treat HBV.

#### Referral Ambivalence

The prospect of antiviral treatment figures ambiguously, alongside the therapeutic power of diet, in Dr. T’s advice to those who test positive:

N.T.: … what do you tell people to convince them that it’s important to do the follow-up…?

Dr. T: Well! *It depends*, eh, it depends … on age … on sex too, it depends on the patients you have. Because there are people who are educated, who know something about it … but for others … you tell them clearly that there is a disease inside you, well, sometimes … it can manifest itself, but *it can also not* … we explain to them, the treatment how it goes, the diet you need to follow … *Especially the diet, because sometimes there is a lack of means, with respect to the correct treatment*…

[…]

N.T.: And you tell them that in some cases it’s possible to treat, that there are medicines…?

Dr. T: Yes, of course, of course! Because there are people even if they haven’t had treatment … *well it’s a treatment*, in quotation marks, who just followed a diet and were ok. Well, I don’t know if it was the test that wasn’t … well or not, but there are people who followed a diet and who came back with a negative test [repeats this several times, as if this is amazing but true]. And, well, those people, we consider them to be cured. There are also people who follow another treatment … an antiviral treatment, who do their viral loads to see the evolution of the disease. There are really advances concerning treatment!” (emphasis mine)

Although he seems to identify antivirals as the “correct treatment,” Dr. T. concedes that this option is not open to all chronic carriers. Conversely, he describes “diet” as effective, but also as a fallback for when “there is a lack of means.” What he is hinting at here, I think, is that he modulates how he communicates the stakes of HBV as part of sorting out candidates for referral for treatment, from the rest, for whom, playing on the uncertainty of HBV effects, he reassuringly insists that the virus may never “manifest” at all and that diet is therapeutic. Another ICP, Dr. P., is more forthcoming about how he tailors his advice:

“You know, when you’re in front of a person, an intellectual, the way of communicating differs from [that] with an illiterate person … you can confuse a person. Us, we know the quality of the person in front of us … with illiterate people … they don’t get nuance, and when you explain certain things, it makes them scared, it terrorises them, they fear death … it’s very complicated!”

His tone here is admittedly patronizing, suggesting doubt in the intellectual as well as emotional capacity of the “uneducated” to handle the implications of HBV infection. But for Dr. P., as for Dr. T., differential ability to “understand” HBV seems to be tangled up with unequal ability to pay for follow-up care. As Dr. P. also put it: “*some* understand very well, and *sometimes* have the means to go get followed up” (emphasizes mine). Dr. D., a former ICP now in private practice, describes himself as the most energetic and successful HBV referrer in the district. He is adamant that persuasive referral depends on conveying just how high the stakes of infection and treatment are: “I tell [them] if you don’t treat, you will have cancer … I don’t mince my words [*je ne lésine pas sur les mots*]!”

These three ICPs are the only PHC workers who told us that they refer at least some HBV positive persons to the regional hospital in Kaolack specifically to be assessed for antiviral treatment. They seem better informed than others: they know treatment is available, but also that it entails frequent travel to the city and expensive tests. Some of their patients may be able to afford this, and, indeed, it is notable that they practice in some of the district’s larger towns, serving populations among which some can be described as members of, or have close connections to, a religious, farming, or political elite. Though none of these ICPs explicitly stated that they referred some but not others, Drs. T. and P. are quite clear that they selectively provide the information by which patients can be *persuasively* referred. This information is not only complex but also, as Drs. P. and D. insist, emotionally charged. By juxtaposing ability to pay for treatment with capacity to understand and handle the stakes of HBV, Drs. T. and P. may be hinting that they judge the latter as a proxy for the former. Yet they may also be implying that informing patients who cannot afford treatment about the potentially fatal outcomes of infection and the availability of lifesaving drugs would *create* a situation of cognitive and emotional incomprehensibility. Selective referral may thus be a manifestation of ambivalence about initiating trajectories into further care amid widespread poverty and lack of communication about HBV.

Ambivalence about referral can also be discerned in midwives’ response to HBV tests. The latter oversee the lion’s share of HBV screening at PHC level. A minority (2 of 11) reported providing *only* dietary advice, without referral, as did a few ICPs. Most midwives, however, described referral to the GP at the district health center in Nioro as standard practice. Yet they are unaware that treatment is available and about the steps required to obtain it. This may limit their motivation and ability to refer *persuasively*, since they cannot tell their patients why, exactly, they should consult the GP. Several stated they felt inadequately trained to deal with HBV infection.^9^ They also suggested the GP would simply confirm the screening test result and reinforce dietary advice. A few thought further testing might be done; indeed, basic tests of liver enzyme function can be performed at district level. None, however, spoke of further referral to the regional level, which is required for treatment eligibility assessment and prescription. At least two doubted the GP referrals they provided were followed-up on. Moreover, all said they told women to wait until after they had given birth to see the GP or put off referring until a postnatal visit. Most midwives also told us their primary concern was to reassure women who tested positive and who, being pregnant, should be protected from strong emotion. They do this by stressing that the virus may remain “dormant” and that following a diet, which they advise starting during pregnancy, can suppress or even clear the infection. My overall impression from midwife interviews was that most referred without much conviction, if at all.

Referral ambivalence, whether enacted as selective referral, nonreferral, or “half-hearted” referral, can be seen as a force of filtration that pushes the majority of HBV carriers away from trajectories into further care and the possibility of treatment. The poor training of health workers as well as the lack of public information about HBV has indeed been identified as a “barrier to linkage to care” in other African settings (Giles-Vernick et al., 2016; Shimakawa et al., 2017). Yet referral ambivalence is also haunted by the prospect of futility that trajectories will be stalled or interrupted, wasting time and money, generating anxiety about the uncertainty of prognosis and the value of care (see Giles-Vernick and Hejoaka, 2020). As Whyte et al. (2004) suggest, there is mutual interaction between unequal access to drugs and broader patterns of socioeconomic inequality. Access may not only reflect ability to afford treatment, but also be shaped by assumptions, for example among health workers, about what care will entail and how it will be understood and prioritized as well as paid for by specific patients. In a way, referral ambivalence can be seen as stemming from an impulse to protect patients from the consequences of unequal access, an impulse that may appear as humane, paternalistic, or unfair. At the same time, it entrenches—particularly when some are selected for referral and not others—existing inequalities in access to resources, knowledge, and care. To understand the reasoning underlying (non-)referral, however, it is important to consider how PHC workers see dietary advice as a form of care.

#### Dietary Self-Care

Regardless of whether or how they refer, nearly all PHC workers report giving dietary advice to those who test positive for HBV. The details vary, but the common thread is to reduce fat intake. Some specify foods to avoid, such as butter, meat, and, most often, peanuts. A few add other “hepatotoxic” substances, notably paracetamol and herbal remedies. For specialists in Europe or Dakar, there is no evidence of *any* effect of dietary restrictions on the outcome of chronic HBV infection. They interpret the widespread “belief” in diet—which appears to cut widely across space and education levels (e.g., Giles-Vernick et al., 2016; Erlinger, 2020; ul Haq et al., 2012)—as the stubborn vestige of now outdated expert opinion. They do, however, recognize an enduring logic: that digestion of overly fatty foods burdens or “tires” the liver, thereby rendering it more vulnerable to infection-related damage.

This is one of the reasons we heard from Nioro PH workers for avoiding fat and oil; these could “accelerate” hepatitis-related disease progression. But we were also told that fatty diets could “cause” HBV *infection,* as could the consumption of aflatoxin-contaminated peanuts. Peanuts are a ubiquitous source of both protein and fat in regional diets, while aflatoxin is the metabolic byproduct of a fungus to which peanut plants and kernels are prone, particularly in Senegal’s climate. For many PHC workers in Nioro, diet is not simply an ancillary measure; they describe it, like Dr. T. did, as a treatment that can keep infected people healthy and in some cases even eliminate the virus altogether. Dietary advice does not therefore seem to be offered merely as a better-than-nothing alternative to referral under conditions of limited knowledge about and access to antiviral treatment.

Dietary efficacy is located, in Nioro, within a dense prognostic and aetiological tangle, where sparse fragments of biomedical evidence (limited screening, rare further assessment, scarce epidemiological data) are projected against experiential knowledge of foodscapes, landscapes, and disease. Let us return to Dr. T.: he did seem to position diet as a lesser and cheaper alternative to antivirals, which he calls the “correct” treatment. Yet he went on to explain that the reason for very high rates of HBV infection in the region was “due to dietary habits, with the use of peanuts, we’ve noticed that people don’t use the good kernels, the good kernels are used for seed, and also for sale. So generally, the bad kernels are used … so naturally in the Saloum [the geographical region] there are many cases [of hepatitis].” By “bad kernels”, Dr. T. means those with signs of damage or mold, indicating they are likely to be contaminated by aflatoxin.

Current biomedical evidence shows that chronic consumption of aflatoxins is, like chronic HBV infection, a risk factor for liver cancer and that both can act in synergy as cofactors (Kew, 2013). Without specifically referring to epidemiological data and aetiological knowledge, most PHC workers in Nioro expressed concerns about pervasive aflatoxin exposure as a cause of liver cancer. Peanuts are the main crop grown in Nioro and a major source of both cash and food. While historically grown for export, a growing portion of the harvest has gone to local consumption and trade since the 1980s or 1990s. Recent regulatory changes along with surplus production have stimulated the growth of domestic commercial sales of kernels as well as oil, paste and flour, which are processed on a small scale in towns and villages (Clavel et al., 2013).

Peanuts saturate Nioro’s landscapes: fields fill the rolling hills; bigger towns are crowded with piles of pods, machines to shell them, warehouses to store them, and trucks to drive them away; the smell of simmering peanuts sauces and roasting kernels and the sounds of pressing and grinding waft along their streets, while piled plastic drums of unrefined peanut oil mark weekly markets; and regional cuisine is made up of a long list of peanut-based dishes. Primary healthcare workers “know” the interaction between peanuts (as fatty or as toxic) and HBV infection not through epidemiological data, but through a juxtaposition of intensities: positive test results and cases of liver cancer alongside the omnipresence of peanuts in the landscape and foodways. As midwife K.—who had hoped, like Dr. T., to organize a communication and screening event—puts it:

Hepatitis is a problem … here … Because Saloum … peanuts, there are a lot here [she repeats this]. So people eat fatty food all the time. All they eat is peanuts. Lunch, dinner, all peanuts. Cooking … *mafe* [a peanut-paste based dish], how many times to they cook *mafe* during the week? *Ceere bi* [millet couscous] they make it [with a peanut sauce], how many times? *Mbaxalou saloum* [a regional specialty made with peanut flour]… Their oil too, it’s made from peanuts. So their whole consumption is based on peanuts. It’s because of this that there is an excessive rate of positive antigens here. Liver cancer, yes, there’s a lot of it.

For many ICPs and midwives, this entanglement underpins the efficacy of dietary management of HBV. For some, a fat- and/or peanut-restricted diet (a few specify further to avoid *bad* peanuts) can slow or halt the damaging effects of chronic infection. This view overlaps, even if it is not perfectly aligned, with biomedical evidence of synergistic relations between aflatoxin and HBV. As mentioned above, emphasizing the efficacy of diet is also a way of reassuring positive individuals, particularly pregnant women. Those who were most emphatic about diet are those, like Dr. T., who say they have seen it reverse antigen test results. Midwife W., who advises patients to avoid peanut paste and paracetamol and to reduce oil and butter, has also seen “women who come back with a negative HBs antigen after, after the diet [she repeats this],” as has Midwife K., who concluded: “so you see the value of educating them in relation, especially, to the diet they have to follow!”

For Nioro’s PHC practitioners, then, access to HBV care is not an “all” (i.e., referral culminating in antiviral therapy) “or nothing” proposition. They may filter a few into further care through selective referral. But others who have been diagnosed as positive are not filtered out of care altogether, even if the dietary treatment offered has limited efficacy on biomedical terms (still, given potential reduction of synergistic interaction between risk factors, may be somewhat protective). A few, like Dr. T., further recommend HBV positive individuals to self-monitor for a prickling sensation in the upper-right abdominal quadrant and sometimes prescribe liver enzyme tests to check for indicators of liver damage, or abdominal ultrasounds (which must be done at regional level), for signs of cancer. These forms of self-care through diet and vigilance are opened up not just by “ignorance” and poor training, but also by the aetiological entanglements of liver disease with peanut-filled diets, the uncertainty and variability of HBV infection outcomes, and lack of access to further diagnostic assessment (and, probably also, also by inaccurate rapid screening tests which may give false positive followed by negative results).

Yet individuals are also filtered into, or out of, dietary self-care. Most midwives noted it was a challenge to get women to pay for prenatal testing. The price of the HBV test was fairly low, at 2,500 CFA/4.4 USD (although it had recently nearly doubled).^10^ It was, however, integrated with a test bundle costing 12,000 CFA/21.1 USD. Midwives complained many could not afford this or that they reported their husbands refused to pay for it. This suggests that poverty combines with gender inequality to filter some out of HBV screening (as well as other tests important to a safe pregnancy and childbirth). There may also be gender, age, and socioeconomic factors of likelihood to donate blood; in Dakar, these include being male, over 40, and attaining higher levels of education (Duboz et al., 2010).

Capacity for dietary change is also unequally distributed. Households in Nioro rely heavily on peanuts and oil (including unrefined peanut oil) as a relatively cheap and abundant source of protein, calories, and taste. Furthermore, eating is a communal process with gendered and generational hierarchies, while meal preparation is time, labor, and fuel consuming. Even the more precise and potentially more useful advice to eat (rather than sell) only “good” peanuts may entail loss of much-needed income. Only those with privileged access to resources—as part of wealthier households and/or because of their position *within* households (see Foley, 2009)—might be able to act on dietary advice. When I pressed ICPs and midwives on the feasibility of cutting out oily foods and peanut products, they usually laughed, indicating that obviously, for a majority of their patients, this was a ridiculous suggestion. Several pointed specifically to gendered constraints: one ICP told me women (the vast majority of those screened) retorted: “well what will I eat then?” Even if they wanted to follow the advice, he explained:

They cannot. And, here in the Saloum, women aren’t really taken into consideration, not really […] So that they can decide absolutely nothing […] Men are the ones who make the decisions. So if you are a homemaker, in your home you say, I’m not going to eat […this or that] you risk having all the problems in the world [he repeats this, for emphasis]!

Another midwife reported a woman being brought in by her family because she refused to eat anything at all after testing positive for HBV. Indeed, for many, the only way of heeding the advice given, mostly, recall, to pregnant women, is to go without. Moreover, self-care turns responsibility for HBV management onto individuals and households (Petersen and Lupton, 1996), and away from claims on collective, or perhaps state, obligations for protection, whether through better food regulation or greater access to diagnosis and drugs. In the end, then, even the lateral expansion of HBV care centered on dietary management generates filtered and therefore stratified access.^11^

### Making Collective HBV

#### Neutralizing Aetiology

The Nioro district lab technician told us of HBV screening activities organized by a village association led by a “very dynamic youth.” Back in Dakar, I met with Saliou, a busy freelance consultant. There were two factors behind the initiative, he told me. First was his own sense of obligation to “do something” in his home village, to which he wanted to maintain his attachment and where expectations were high given he obtained a Ph.D. from a North American university and his father played an important role in national politics. Not wanting to go into politics, as village elders pressed him to, he opted to launch a “citizen action movement” which would work in various domains, including health. The second factor (he had not lost the thread of his two-part structure even after a half-hour of talking and eating), was an intense, cumulative experience of deaths in the village due to what some labelled liver cancer. “There is not a single house[hold] in the village that hasn’t lost a young person [to the disease],” he told me. This triggered not only grief, but also pervasive fear (a “psychosis”) and divisive accusations of witchcraft. He recounted asking himself: “Will we let this disease destroy us? Let inaccurate beliefs dictate our actions?” By organizing conferences about HBV and offering screening tests, which began in 2017, the movement would thus recast the deaths as arising from HBV infection that was highly prevalent in the village and a cause of liver cancer.

The purpose of raising HBV “awareness” in this village, which I will call Keur Laye, was, as in PHC settings, not primarily to launch trajectories toward further diagnostics and antiviral drugs. As in the health posts, those found positive in Keur Laye were reassured their diagnosis was not “synonymous with liver cancer” and were given dietary advice. In the first year, Saliou also paid for liver enzyme testing. But in addition to opening up this space of lateral (or merely minimal) posttest care, HBV knowledge in Keur Laye was valued for establishing new causal explanations for a shared history of misfortune, thereby shifting attributions of responsibility in a collective “moral imagination” (Livingston, 2005). In this final section, I turn to the intended effects, particularly on understandings of shared risk and responsibility, of HBV knowledge distribution, first in Keur Laye, and then in the work of patient advocate Ibrahima Gueye (who was also one of the speakers invited to Keur Laye).

Aissatou Diouf and I went to Keur Laye to meet with members of the movement. Gathered in a circle in a courtyard at dusk, they described how the repeated deaths of mostly young men, occurring after rapid weight loss and abdominal swelling, had affected this village of about a thousand inhabitants. As far as he could remember, said the eldest of the group, more than forty had died since 1976, others said one or two every year. Most of the victims were men, and all were young, in their twenties and thirties, so their deaths “really hurt.” Members of the movement were also young men. They spoke of the blood drive (the first screening session having been organized as such to qualify for free testing and reduce stigma) as an “awakening.” Before was a time of ignorance, when recurring illness and death were attributed to possession or evil eye, and there was a lot of “fighting” (which I suspect is an understatement) in the village. With the blood screening, “many cases were revealed, that’s when we knew that it is hepatitis that brought this problem.” Or, as another put it: that all this time, it was “just hepatitis.” Back in Dakar, Saliou had told me (he was not in Keur Laye that evening) villagers had come to him after Gueye’s well-attended conference to say they felt “relieved of a pressure. The situation had been real tense because of the disease.” “The HBV initiatives had succeeded,” he suggested, because they had managed to “demystify, to render banal [*banaliser*] the disease.”

The young men of Keur Laye were not the first to tell me of the association between liver disease and witchcraft accusations. Former heads of medical districts in Dakar, as well as several Nioro ICPs, explained that deaths occurring after rapid wasting and abdominal swelling were often attributed to someone—often a jealous woman or witch—having given the victims “something to eat” in order to take possession of them. Occult aetiologies for similar symptoms have also been noted by anthropologists in other regions of Senegal (Foley, 2009; Boye et al., 2020). The health workers I spoke to, in Nioro and Dakar, worried about these witchcraft accusations not because they saw them as unscientific, but due to their consequences: wasted money on divination, sacrifices, and remedies; consumption of remedies meant to expel the ingested occult substance, but which instead accelerated disease progression; and above all the durable divisions and tensions that such accusations kindled within and between households: “It dislocates relations … dislocates families!,” exclaimed one former ICP, who told us of tensions within his own family that persisted years after his mother’s death from liver cancer. Another ICP recounted a case in which the accused—the wife of the victim’s best friend—had been beaten and locked up with the victim. The ICP had intervened, giving the accusers a “sermon” about the diagnosis of liver cancer, after which the case was “settled amicably” through monetary compensation and divorce.

Members of the movement described HBV screening as successful in neutralizing a collective causal narrative around deaths, thereby alleviating the tensions that had arisen from occult and interpersonal explanations. Yet they also admitted that knowing about HBV, and one’s status, was not easy. Saliou told me that, initially, a “rival” group had discouraged people from getting tested, calling his movement “irresponsible” for “not doing anything” for those diagnosed as positive. Others also spoke of the difficulty of following dietary advice. One asked poignantly how, when he could barely cover household expenses, he could help his HBV positive wife stay healthy. Probably because they hoped I might help mobilize resources, but perhaps also because the recurring deaths and information/screening sessions had led them to frame HBV as a *collective affliction*, members of the group emphasized the need for—even a sense of entitlement to—outside help. In other words, they rejected an individualization of responsibility for HBV self-care. Yet the help they asked for was for good food, not for further diagnosis or drugs.

Saliou, however, was troubled by the knowledge, albeit vague, that with greater resources he and his movement might be able to offer more, biomedically, to those screened as positive. Ibrahima Gueye, he said, had “brought treatment up, but not in detail” during his conference in Keur Laye, so Saliou was unsure of what exactly further care would entail. The high cost of this care seems to make antiviral treatment practically unmentionable in many settings, even during HBV awareness-raising and screening activities. Both Saliou and Gueye blame the state for limits and gaps in HBV care and communication. Calling the state “irresponsible,” Saliou exclaimed: “what we are doing, it’s the government that should be doing it!”

#### An Exposed Nation

Ibrahima Gueye has called for greater state subsidization of HBV care, particularly of diagnostic tests, including, recently, free screening (Diatta, 2018). Yet I never heard him framing access to cheaper, free, or public HBV care, including treatment, as a *right* (human, civic or otherwise). We met several times during my fieldwork; I also heard him intervening in a research symposium and collected newspaper articles and YouTube videos of his media presence. My overall impression was that he brings up the need for more “awareness raising” [*sensibilization*] about HBV more often, and with greater emphasis, than that for greater *access* to care. Much of his advocacy work, with other members of *Saafara Hépatites* (of which he is the nearly exclusive public face), focuses on screening and information. This includes World Hepatitis Day, conferences in villages and in prisons (which Gueye was doing in 2019 in collaboration with a prisoner welfare NGO), and newspaper and television interviews, in which Gueye emphasizes the scale of exposure in Senegal and the need to get tested.

Gueye’s efforts thus seem to work *within,* rather than against, a topography of unequal access to largely privatized HBV care. By informing people about the risk they face and what they can do about, more may decide to pay for care. He insists, for example, on the possibility of vaccination for those who test negative. This is a reason he gives for why even those who cannot afford specialized care should get tested. A course of three vaccine doses for adults is subsidized and costs 5,000 CFA/9 USD (infant HBV vaccination is free). The epidemiological logic of adult vaccination is debatable, given low rates of susceptibility in Senegal. Epidemiological data indicates that most adults who test negative for HBsAg antigen are already immune (e.g., Coursaget et al., 1993). However, antibody testing is more expensive than vaccination, so many Senegalese specialists recommend the latter as potential protection regardless of immune status. Getting vaccinated as an adult is, in both epidemiological and economic terms, a private endeavor. “Yes, that’s a bit expensive,” Gueye admitted of the vaccine price, “but if people are well informed, they can pay. It costs less than this watch, this phone, this dress…” he went on, pointing to objects around us. Similarly, on a Dakar-based YouTube channel (Yesdakar, 2019), he said: “some people will say I don’t have 5,000 for the test, I don’t have 5,000 for the vaccine, but we pay 150,000 for a phone…”.

Gueye’s emphasis on willingness to pay for *relatively* affordable HBV screening tests and vaccines may index a more general acceptance of (or resignation to) the privatization of HBV care and resulting inequalities. “Personally,” Gueye told me, “I’m against free care [*la gratuité*]. Subsidization, sure, but there has to be a minimal price … there’s always someone who pays, who will pay tomorrow … people get used to it.” I heard specialists speak similarly about charging for antiviral drugs. Desclaux (2004) describes how the initial design of Senegal’s HIV treatment initiative rested on assumptions—among both local professionals and entrenched in international health policies—about the inherent value of user fees, which would foster a sense of “dignity” as well as responsibility (translating as adherence) among patients and activate “traditional solidarity networks.” The acceptance of user fees for HBV care may similarly reflect a broader “internalization” of the logics of the health reforms initiated under structural adjustment, whereby only the most cost-effective mass measures such as infant vaccination can count as public goods, and other care is either dispensed as “charity” or at least partly privatized by cost sharing (see, e.g., World Bank, 1993; Foley, 2009). Intensified global health investments in the mid-2000s, along with demands for care as a *right* (as HIV treatment was reframed, Desclaux, 2004), have expanded the scope of public health—but HBV care continues, as Sall Diallo often points out, to be excluded from this scope. Discussions about access continue to revolve around affordability; that is, *how much* “users” will pay rather than *who* should bear the price of care (and who may profit from it, for example, in the commercial economy of testing equipment, supplies, and services).

While Gueye’s “awareness-raising” individualizes responsibility for care, it also seeks to deindividualize and destigmatize responsibility for infection by insisting on the collective nature of *exposure*. He likes to illustrate this point by evoking an image familiar to many Senegalese adults of schoolchildren lined up to be vaccinated with a jet-gun. As the host of a 2012 talk show laughed, presumably at her own memory of this image, Gueye pressed on: “one single needle, five hundred people […] the reason I bring this up [is to emphasize that] hepatitis, it concerns us all, everyone is at risk” (Senewebdirect, 2012). To me, he said, “I show the scar on my arm. People see it and tell themselves they too might be affected.” Sall Diallo also points to widespread risk; “hepatitis concerns us all” was a slogan she circulated, along with the figure of an 85% exposure rate (i.e., nearly universal contact resulting in immunity or infection. Others, such as Coursaget et al., 1993, put it at over 90%). Nevertheless, PNLH declarations and activities have emphasized “risk groups” such as health and sex workers.^12^ Gueye refuted this on television: “the *whole population* is at risk, the numbers show it!” (2STV 2019)

Sall Diallo appears unworried about stigmatizing HBV; for example, she frequently and bluntly reminds audiences that sex is a mode of transmission. By contrast, Gueye treats sexual transmission as a delicate issue. He explained his strategy to me:

I cannot be said that it does not exist. It can exist. But I bring it up last, starting upstream. When someone is positive, they cannot know when they were infected. The first possibility is that they were born with it. That’s to reassure […] for the majority here in Africa, that’s it. In any case, it lifts a weight. I summon the past first.

Evoking uncertainty about infection source, early-life transmission, and serial childhood vaccination are, for Gueye, ways of conveying HBV as a neutral and widely shared exposure; a risk for which individuals cannot be held responsible. This is a strategy to counter stigma and the kinds of tensions he has witnessed around HBV diagnoses: for example, of men seeking to cast out their infected wives. His goal, he states, is “that the person does not feel responsible.” Gueye sees stigma as an obstacle to both (individualized) care-seeking and collective mobilization.

The work of Keur Laye’s movement and of Gueye and *Saafara Hépatites* communicates to audiences that HBV circulates widely among them and that they should not be held responsible for their status, nor should they accuse each other of transmission or of causing swollen-stomach deaths. HBV knowledge is treated as having the power to reconstitute social relations around shared infection, risk, disease, and loss. In neither case has this emergent sense of HBV as a collective burden been explicitly linked to arguments for redistributing the costs of care through collective, public mechanisms. Yet the potential is there: reframing HBV as collective misfortune, in which some must bear the bodily effects of its variable outcomes but should not necessarily be made to bear the financial and logistical costs of mitigating these, may serve as a basis for making claims to free and public care as a right.

## Conclusion

Further research is needed to determine whether and how clinical interactions, as well as other modes of communication about HBV, may filter individuals in or out of care and thereby mediate access inequalities. My research has been limited to what actors involved in the provision of HBV information and care *say* about what they do and why. There is more to be learned through observation of clinical and educational practices and by tracking their effects on patients and audiences, as well as on trajectories of testing and care (likely in combination with information-sharing and decision-making among kin networks). Yet my focus, via HBV actors, on the topography of specialized care and HBV communication, alongside screening and information efforts that largely fail to join up with this topography, opens up a vista onto uneven provisions of *both* HBV technologies and knowledge and a glimpse of interactions between them. This has allowed me to identify filtration—which arises from these interactions—as a mechanism that produces inequalities in access to care and, at the same time, renders these inequalities less visible and less open to contestation.

By attending to the indirect effects of access inequalities on enactments of HBV, I have sought to illuminate complex entanglements among HBV knowledge/communication, “means” (to pay for care), privatization, gendered and socioeconomic disparities, explanatory models of causation and efficacy, and assumptions about who can and should bear the costs of care. Access is not determined only by who knows about, or can pay for, what kind of care. “Filtration” describes this nonlinear, dynamic entanglement by which different sites and mechanisms of inequality are mutually enacted and constitute—or not—potential subjects of HBV care.

To conclude, I want to highlight two themes amid this dense tangle: privatization and gender. HBV has been pointed to as a neglected issue in global health (e.g., Lemoine et al., 2012) despite its heavy burden of morbidity and mortality. My research suggests this neglect, at the level of what PNLH director Sall Diallo calls “global health governance,” which gets reproduced in national healthcare policy and practice,^13^ hinders not just action on, but even the articulation of, HBV as a *public* health issue. For one, there are few resources to detect and communicate the scale of infection at the national level and thus frame it as a collective problem. In addition, the distribution of scarce resources for care both assumes and reinforces private responses to (the risk of) infection and illness. Infected individuals are expected to pay, in part or in whole, for diagnostics, drugs, or “therapeutic” diets. The provision of most of these services, as well as communication about HBV, have been left to personal and/or commercial initiatives, with little or no public oversight. Even the nominally public but underfunded PNLH manifests as a highly personalized presence. This results in uneven and fragmented distributions of both HBV care and information about it, so that subjects of treatment are formed in spaces of privileged access that remain largely invisible and uncontested. Moreover, widespread emphasis on personal responsibility for exposure (or at least, a lack of effort to *deemphasize* risk behaviors such as sex) and for care, including self-care, deflects attention from potential collective models of viral circulation and protection. There are sites of tentative conceptualizations of HBV as a shared problem that should be tackled collectively through public channels, but these have yet to give rise to vocal demands for access to treatment.

The privatization of HBV and its care partly overlaps with its gendering. As the PHC practitioners we interviewed point out, expectations that individuals can and should pay for HBV screening tests and that dietary restriction is an effective and accessible form of self-care, are both challenged by and reinforce gendered household dynamics. More research is needed on the gendered implications of focusing screening efforts on pregnant women, especially given widespread assumptions about the sexual transmission of HBV. Gueye, for example, has hinted that diagnoses of HBV often provoke suspicion, rejection, guilt, and confusion due to these (unfounded) assumptions. Yet epidemiologically validated emphasis on perinatal and early childhood HBV exposure as both frequent and risky (more likely to lead to cirrhosis and cancer) also draws attention to mothers as transmitters of an infection that tends to kill more men. How do HBV data and models shape understandings of gendered relations of care, pleasure, and harm? Similar questions can be asked of occult forms of swollen-belly death: in all the stories I heard, the accused were always—often jealous—women.^14^

Points and processes of filtration—whether as orientation into lateral care (diet or nonbiomedical healers), unpersuasive referrals or too-expensive, unexplained test prescriptions—arise from *partial* expansions of access to diagnosis and drugs. Increasing the availability of screening tests, viral load testing or antivirals are likely to have unintended effects if not accompanied by a *public* strategy for their coordination, and the fair distribution of resources, including information, and costs. A focus on filtration, rather than on the proportion of treatable individuals getting treatment, provides a fuller and more nuanced view of what happens in the gap between the availability and accessibility of biomedical technologies.

## Data Availability

The datasets presented in this article are not readily available because interview content may include personal or identifiable data even if anonymized. Requests to access the datasets should be directed to n.tousignant@ucl.ac.uk.

## Footnotes

1 Blood for transfusion has been screened in Senegal since 1982 (Programme National de Lutte contre les Hépatites, 2018).

2 Specialists complain about “ignorance” among lower-tier health workers, while some of the latter, I have found, report feeling inadequately trained. I heard of (and from) persons diagnosed as HBV positive who were told there was not biomedical treatment for HBV and referred for nonbiomedical care or, as will be detailed below, were given only dietary advice. Similar findings are reported for Burkina Faso by Giles-Vernick et al. (2016).

3 Lamivudine was the first reverse-transcriptase inhibitor which, after being routinely used in HIV treatment, was approved for the treatment of HBV (by the FDA in 1998). It was welcomed as a significant improvement over pegylated interferon, which was only effective in some patients, administered by injection and reputed for painful side effects.

4 Tenofovir disoproxil fumarate, initially commercialized as Viread, was approved by the FDA to treat HIV in 2001 and to treat HBV in 2008. Many patients treated with lamivudine developed drug-resistant HBV infections, so tenofovir was quickly adopted as the drug of choice.

5 One hospital specialist told me, however, some patients presented with clinically evident cirrhosis and could thus be put on free antiviral therapy without further testing.

6 The same document reports national prevalence rates of chronic infection at 9–11% (out of a population of about 15 and a half million). Even if only 5–10% of carriers require treatment, this suggests that only a tiny portion of these—or indeed, of those who test positive every year through blood donation screening (8,757 in 2017)—are accessing it.

7 By contrast, HIV/AIDS control received 10–14 billion CFA per year in 2013–2018, of which about a third was managed by the national AIDS program (and a quarter to a fifth contributed by the Senegalese state, the rest made up of donor funding) (annual reports available on: https://www.cnls-senegal.org). Budgets for malaria control were of 18 billion CFA for 2016 and nearly 13 billion for 2017 (http://www.pnlp.sn/wp-content/uploads/2016/08/PNLP_PSN_VFF_03-02-2016.pdf).

8 Some ICPs, however, did not report administering HBV tests or advising carriers.

9 Midwives were trained to administer birth dose HBV vaccine, which was introduced in 2016, but many said they were not taught to emphasize vaccination for babies of those who tested positive.

10 Testing kits could also, according to Gueye, be procured at a much lower cost. Most health posts did not have testing kits, even though tests used at the district level are suitable for point-of-care testing.

11 Anthropologists of HIV treatment programs have also noted that access to food, even when drugs are provided for free, becomes a site of treatment inequality, given that patients are educated that they must eat well in order for ARV treatment to work effectively. See, e.g., Kalofonos (2010), Prince (2012).

12 I heard other Senegalese experts speak of risk groups as well as sexual, iatrogenic, and parenteral transmission among adults. Others, however, assert that infection is distributed throughout the “general” adult population, while epidemiological data suggest that sexual transmission is absent or negligible given pervasive childhood exposure to HBV in Africa.

13 This happens in both direct ways, through lack of donor funding for HBV action, and indirect ways, when as national priorities are set to capture available resources.

14
Livingston (2005) notes that women were also often accused of responsibility for children’s disabilities in Botswana. Elsewhere in Africa, witchcraft accusations have often been linked to tensions in gendered roles and relations (e.g., Drucker-Brown, 1993).
